The article "Effect Evaluation of Platelet-Rich Plasma Combined with Vacuum Sealing Drainage on Serum Inflammatory Factors in Patients with Pressure Ulcer by Intelligent Algorithm-Based CT Image" was retracted in 2023. Reasons: signs of a paper mill; compromised peer review; unreliable results or conclusions.

# Effect Evaluation of Platelet-Rich Plasma Combined with Vacuum Sealing Drainage on Serum Inflammatory Factors in Patients with Pressure Ulcer by Intelligent Algorithm-Based CT Image

**DOI:** 10.1155/2022/8916076

**Published:** 2022-03-02

**Authors:** Jingzhe Yang, Changshuan Xiao, Hailing Wen, Kui Sun, Xiaoming Wu, Xinshu Feng

**Affiliations:** Department of Burn and Plastic Surgery, Affiliated Hospital of Chengde Medical University, Chengde, 067000 Hebei, China

## Abstract

This work was to explore the efficacy of intelligent algorithm-based computed tomography (CT) to evaluate platelet-rich plasma (PRP) combined with vacuum sealing drainage (VSD) in the treatment of patients with pressure ulcers. Based on the u-net network structure, an image denoising algorithm based on double residual convolution neural network (Dr-CNN) was proposed to denoise the CT images. A total of 84 patients who were hospitalized in hospital were randomly divided into group A (without any intervention), group B (PRP treatment), group C (VSD treatment), and group D (PRP+VSD treatment). Procalcitonin (PCT) was detected by enzyme-linked immunosorbent assay (ELISA) combined with immunofluorescence method, C-reactive protein (CRP) was detected by rate reflectance turbidimetry (RRT), and interleukin-6 (IL-6) was detected by electrochemiluminescence method. The results showed that after treatment, 44 cases (52.38%) of pressure ulcers patients recovered, 24 cases (28.57%) had no change in stage, and 16 cases (19.04%) developed pressure ulcers. The pain scores of group D at 1 week (3.35 ± 0.56 points) and 2 weeks (2.76 ± 0.55 points) after treatment were significantly lower than those in group C (7.77 ± 0.58 points and 6.34 ± 0.44 points, respectively). The time of complete wound healing in group D (24.5 ± 2.32) was obviously lower in contrast to that in groups A, B, and C (35.54 ± 3.22 days, 30.23 ± 2 days, and 29.34 ± 2.15 days, respectively). In addition, the medical satisfaction of group D (8.74 ± 0.69) was significantly higher than that of groups A, B, and C (4.69 ± 0.85, 5.22 ± 0.31, and 5.18 ± 0.59, respectively). The levels of IL-6 and PCT in group D were lower than those in groups A, B, and C, and the differences were statistically significant (*P* < 0.01). The average values of peak signal to noise ratio (PSNR) and structural similarity index measure (SSIM) of the Dr-CNN network model were 37.21 ± 1.09 dB and 0.925 ± 0.01, respectively, which were higher than other algorithms. The mean values of root mean square error (MSE) and normalized mean absolute distance (NMAD) of the Dr-CNN network model were 0.022 ± 0.002 and 0.126 ± 0.012, respectively, which were significantly lower than other algorithms (*P* < 0.05). The experimental results showed that PrP combined with VSD could significantly reduce the inflammatory response of patients with pressure ulcers. PRP combined with VSD could significantly reduce the pain of dressing change for patients. Moreover, the performance model of image denoising algorithm based on double residual convolutional neural network was better than other algorithms.

## 1. Introduction

Pressure ulcer, also known as bedsore, is an ulcerated necrosis of the skin caused by local tissue hypoxia, insufficient nutrition, and lack of nutrition due to pressure, which is a common complication in clinical practice [1, 2]. There are many causes for the formation of pressure ulcer, such as long-term bed rest, paralysis, diabetes, or vascular disease after surgery. However, with the development of society and the process of population aging, the incidence of a series of chronic diseases such as diabetes and hypertension is increasing year by year, which also accelerates the occurrence of pressure ulcer [3–5]. Pressure ulcer is generally divided into congestion ruddy stage, inflammatory infiltration stage, superficial ulcer stage, and necrotic ulcer stage [6]. How to effectively prevent and treat it has always been a problem to be solved, and many scholars have also devoted themselves to solving it for many years [7].

Clinically, the common treatments are vacuum sealing drainage (VSD) and platelet-rich plasma (PRP) [8]. The principle of VSD treatment is to improve the local blood circulation of the wound and remove necrotic tissue by vacuum aspiration, thereby accelerating the proliferation of granulation tissue and reducing tissue edema [2, 4]. PRP is a platelet concentrate containing growth factors and cytokines extracted from its own peripheral blood, and it was found that this method can effectively promote tissue nerve repair and angiogenesis, achieving significant efficacy in the treatment of chronic refractory wounds [9, 10]. The mechanism of action of PRP is to regulate inflammation by reducing the levels of IL-1*β*, which can release a large number of growth factors, such as epidermal growth factor and vascular endothelial growth factor, which can promote cell proliferation so as to achieve the purpose of repairing the wound and accelerating healing [11, 12]. Although the clinical use of the two is common, there are few reports on the combined use of the two to treat the disease [13].

Most of the pressure ulcer patients initially have local skin and soft tissue defects on the sore surface, and it is impossible to determine the lesions of the surrounding tissue, resulting in the sore surface often protracted and unhealed. With the improvement of modern science and technology, computed tomography (CT) imaging technology is widely used to assist doctors in the diagnosis of pressure ulcers. However, when the X-ray tube current is reduced in the process of CT imaging mechanism, the number of photons reaching the detector is greatly reduced, and the generated quantum noise seriously affects the imaging effect [14–16]. The appearance of these noises greatly reduces the quality of images and causes a visual impact on clinicians, which affects the diagnosis and treatment of diseases. Deep convolutional neural networks are widely used in image analysis. However, with the increase of network depth, in the process of convolutional neural network (CNN) training, it is easy to have too many gradients or disappear, so that the training cannot be carried out normally. This resulted in a deep residual network that alleviated the network training problem by adding residual learning units to the convolutional layers [17]. At present, deep residual networks have been widely used in the optimization of medical images.

In summary, how to effectively prevent and treat pressure ulcer remains to be solved. PRP and VSD have good effect in the treatment of refractory wounds, and deep residual network can effectively deal with the noise problem in CT imaging. Therefore, this study proposes a CT image noise reduction algorithm based on double residual convolution neural network (Dr-CNN) model for evaluating PRP combined with VSD treatment in pressure ulcer, in order to improve the theoretical support for the use of deep learning technology in imaging and clinical treatment.

## 2. Materials and Methods

### 2.1. Research Objects

A total of 84 patients (48 males and 36 females, aged 22-72 years) with pressure ulcer in hospital from June 2017 to December 2020 were selected as the research objects. All patients were divided into four groups according to the random number table, with 21 patients in each group: group A (without any intervention), group B (PRP treatment), group C (VSD treatment), and group D (PRP combined with VSD treatment). General clinical data of patients were collected in the study, and all patients underwent CT examination. This study has been approved by medical ethics committee of hospital, and the patients and their families understood the study and signed the informed consent form.

Inclusion criteria were defined as follows: (I) patients with pressure ulcers who had no healing tendency after regular treatment for more than 1 month; (II) age ≥18 years old; (III) patients without major organic diseases, diabetes, burns, etc.; and (IV) patients with complete clinical data.

Exclusion criteria are as follows: patients with poor compliance; patients with unstable vital signs; patients combined with severe cardiopulmonary disease; patients with contraindications to CT examination; patients with neurological dysfunction; and pregnant women.

### 2.2. Treatment Methods

#### 2.2.1. Group A

Routine disinfection, debridement, thorough cleaning of local necrotic tissue, abscess, and foreign body, with hydrogen peroxide solution (500 mL/bottle), iodophor, and saline were used to repeatedly rinse the wound, according to the exudation of dressing, dressing change every 2 to 3 days, and necrotic tissue and abscess were cleaned timely.

#### 2.2.2. Group B

Based on group A, group B was combined with PRP treatment, and 10-15 mL peripheral venous blood of patients was collected and placed in an anticoagulant sterile centrifuge tube for secondary centrifugation. The first centrifugation (2,500 r/min, 10 min) was performed. After it was divided into three layers, the supernatant was taken out and placed in another centrifuge tube. After centrifugation again (2,500 r/min, 10 min), after it was divided into two layers, 3/4 of the supernatant was taken out, and the rest was PRP. Then, the obtained PRP was mixed with thrombin-calcium mixture according to 10: 1 to form platelet-rich gel. According to the doctor's advice, platelet-rich gel was evenly dripped on the wound of pressure ulcers, which was wrapped with sterile gauze, once every three days.

#### 2.2.3. Group C

Based on group A, group C was combined with VSD treatment, according to the depth and length of drainage wound, shape, etc., and the dressing was prepared and cut to the shape of the wound. The dressing was placed on the wound. After the drainage tube was placed, the dressing around the wound and the drainage tube were sealed and wrapped with semipermeable membrane. The other end of the drainage tube was connected to the negative pressure suction device, and the parameters were set according to the specific conditions of the wound. Attention was paid to the observation of the drainage to ensure smooth drainage.

#### 2.2.4. Group D

Based on group A, patients were treated with combination of group B and group C.

#### 2.2.5. CT examination

Spiral CT scanner was used for CT examination; parameter settings are as follows: matrix: 512 × 512; layer spacing: 5 mm; layer thickness: 5 mm; and through the current: 200 mAs; and cross-sectional plain scan was performed.

### 2.3. Dr-CNN Network Model

In order to reduce the loss of projection data in CT imaging and solve the overfitting problem, the projection domain network, domain conversion layer, and image domain network were integrated in this study, and the Dr-CNN network model was designed. This model was divided into three parts: projection domain part, domain conversion part, and image domain part (Figure 1).

It is assumed that *m* ∈ *H*_1_ represents the original data of low-dose CT imaging, and *n* ∈ *H*_2_ represents the data of normal-dose CT imaging of this image. The noise reduction learning can be a function *K*_1_ of *m* mapping to *n*, which can be expressed as follows.

(1) $$\begin{array}{c} K_{1}:m⟶n. \end{array}$$

The FBP module is used as the domain conversion instead of the full connectivity layer, and the output of the projection domain subnet is decoded into a CT image with low signal-to-noise ratio, which can be expressed as follows.

(2) $$\begin{array}{c} C:K_{1}\left(m\right)⟶C\left(K_{1}\left(m\right)\right). \end{array}$$

*C*(*K*_1_(*m*)) is the CT image with low signal-to-noise ratio obtained after *K*_1_(*m*) transformation by FBP noise reduction processing. In order to reduce the error, the image domain part can be expressed as follows.

(3) $$\begin{array}{c} K_{2}:C\left(K_{1}\left(m\right)\right)⟶C\left(n\right). \end{array}$$

*C*(*n*) means the normal dose CT imaging of this image. The Dr-CNN network structure can also be divided into three parts: projection domain subnetwork, domain conversion, and image domain subnetwork (Figure 2). Mean square error (MSE) is usually used as the objective optimization function in low-level image processing tasks. Therefore, in this study, the objective function is divided into two parts, which can be expressed in Equation (4).

(4) $$\begin{array}{c} S=\lambda_{1}V_{E}\left(K_{1}\left(m\right),n\right)+\lambda_{2}V_{Q}\left\{K_{2}\left(C\left(K_{1}\left(m\right)\right)\right),C\left(n\right)\right\}. \end{array}$$

*K*_2_(*C*(*K*_1_(*m*))) indicates that the image with high signal-to-noise ratio processed by the subnetwork of image domain can be regarded as normal-dose CT image. *V_E_* and *V_Q_* represent the MSE loss in the projection domain subnet and the image domain subnet, respectively. *λ*_1_ and *λ*_2_ denote the balance coefficients to be learned in the projection domain subnet and the image domain subnet, respectively. All training and testing tasks in this study were performed on a TensorFlow deep learning framework with a single GPU (NVIDA TITANV, 28 GB memory).

### 2.4. Observation Indexes

Procalcitonin (PCT) was detected by enzyme-linked immunosorbent assay (ELISA) combined with immunofluorescence method, C-reactive protein (CRP) was detected by rate reflectance turbidimetry (RRT), and interleukin-6 (IL-6) was detected by electrochemiluminescence method. Wound healing, patient pain score, wound healing time, and satisfaction were also recorded.

Image quality evaluation indicators were as follows.

The filtered back projection (FBP) reconstruction algorithm [18], total variation minimization (TV algorithm) [19], and block-matched three-dimensional filtering (BM3D algorithm) [20] were introduced. The normalized mean absolute distance (NMAD), root mean square error (RMSE), structural similarity index measure (SSIM), and peak signal to noise ratio (PSNR) were compared to evaluate the noise reduction effect of the model.

(5) $$\begin{array}{c} NMAD=\frac{\underset{x=1}{\overset{G}{\Sigma }}\left|n\left(x\right)-m\left(x\right)\right|}{\underset{x=1}{\overset{G}{\Sigma }}\left|n\left(x\right)\right|}, \end{array}$$

(6) $$\begin{array}{c} RMSE=\sqrt{\frac{\left(\underset{x=1}{\overset{G}{\Sigma }}{\left|n\left(x\right)-m\left(x\right)\right|}^{2}\right)}{N}}, \end{array}$$

(7) $$\begin{array}{c} PSNR=10\log_{10}\left[\frac{MAX^{2}\left(n\right)}{\left(1/N\right)\left(\underset{x=1}{\overset{G}{\Sigma }}{\left|n\left(x\right)-m\left(x\right)\right|}^{2}\right)}\right]. \end{array}$$

*m* represents the final reconstructed image, *n* represents the true value image, *x* represents the index value of the image, and *G* is the total number of pixels.

(8) $$\begin{array}{c} SSIM\left(P,Q\right)=\frac{\left(2\alpha_{P}\alpha_{Q}+G_{1}\right)\left(2\rho_{PQ}+G_{2}\right)}{\left(\alpha_{P}^{2}+\alpha_{Q}^{2}+G_{1}\right)\left(\rho_{P}^{2}+\rho_{\text{Q}}^{2}+G_{2}\right)}. \end{array}$$

*P* is the original image, *Q* represents the image to be compared, (*α*_*P*_, *α*_*Q*_) represents the brightness of image, (*ρ*_*P*_, *ρ*_*Q*_) represents the contrast of image, and *ρ*_*PQ*_ is the structure of image.

The higher the PSNR value of the index is, the closer the reconstructed image is to the reference image visually; the lower the values of NMAD and RMSE, the smaller the difference between reconstruction results and ideal results, and the better the image quality. The SSIM index comprehensively measures the similarity between the reconstructed image and the reference image from the three aspects of contrast, brightness, and structure retention. The closer the SSIM value is to 1, the closer the reconstructed image is to the real image.

### 2.5. Statistical Analysis

The data processing of this study was analyzed by SPSS 19.0 statistical software. The measurement data were expressed as mean ± standard deviation ($\overset{¯}{\text{x}}\pm \text{s}$), and the enumeration data were expressed as percentage (%). One-way analysis of variance was used for pairwise comparisons. The difference was statistically significant at *P* < 0.05.

## 3. Results

### 3.1. Noise Reduction Performance of Dr-CNN Network Model

The noise reduction performance indicators of the four algorithms were compared, and the results were given in Figure 3. The mean values of PSNR and SSIM of Dr-CNN network model were 37.21 ± 1.09 dB and 0.925 ± 0.01, respectively, which were higher than those of LDCT, TV, and denoising convolutional neural network (DNCNN); the mean values of RMSE and NMAD of Dr-CNN network model were 0.022 ± 0.002 and 0.126 ± 0.012, respectively, which were significantly lower than those of other algorithms, and the differences were statistically significant (*P* < 0.05). It shows that the Dr-CNN network model has better stability and noise reduction effect.

In addition, the average running time of the four algorithms was also compared, and the results were illustrated in Figure 4. It was found that the time for the Dr-CNN network model to process a figure may be related to the complexity of the algorithm results and the parameter counts.

### 3.2. Comparison of Noise Reduction Effect of Four Algorithms

Figure 5 showed the CT image of deep tissue pressure injury at the sacrococcygeal region of a 53-year-old male patient.  Figure 5(a) was the original image, and Figures 5(b)–5(e) indicated the noise reduction results of LDCT, TV, DNCNN, and Dr-CNN algorithms, respectively, which suggests that Figure 5(e) is the clearest and has the best noise reduction effect.

### 3.3. Comparison of General Clinical Data of Patients

The general clinical data of the four groups were statistically analyzed and compared. The results showed that there was no significant difference in gender, age, and grade among the four groups (*P* > 0.05), indicating the feasibility of the experiment (Figure 6).

### 3.4. Statistics of Treatment Results

In the 84 subjects, 44 cases (52.38%) recovered after treatment, 24 (28.57%) had no change in stage, and there were 16 (19.04%) occurrence of pressure ulcer (Figure 7).

### 3.5. Pain Score

The pain scores of the four groups before surgery, one week after surgery, and two weeks after surgery were statistically analyzed, and the results were given in Figure 8. There was no significant difference in the preoperative pain scores among the four groups, without statistical significance. After surgery, the pain scores of groups B, C, and D were significantly lower than those before surgery, and the difference was statistically significant. Moreover, the postoperative pain score of group D was significantly lower than that of other groups, and the differences had statistical significance (*P* < 0.05). It reveals that the conventional treatment is not effective in relieving the pain of patients. Although the use of PRP or VSD can relieve the pain, the effect is less than the combination of the two.

### 3.6. Comparison of Postoperative Wound Healing Time

The time of complete wound healing in the four groups after operation was 35.54 ± 3.22 days, 30.23 ± 2 days, 29.34 ± 2.15 days, and 24.5 ± 2.32 days, respectively. As shown in Figure 9, the time in group D was significantly shorter than that in groups A, B, and C, and the difference had statistical significance (*P* < 0.05). The use of PRP combined with VSD can effectively shorten the wound healing time of patients.

### 3.7. Comparison of Serum Inflammatory Factors

The serum inflammatory factors of four groups of patients before and 20 days after surgery were compared, and the results were shown in Figure 10. There was no significant difference in the mean CRP (mg/mL), PCT (pg/mL), and IL-6 (ng/L) values of the four groups of patients before surgery. Postoperative CRP, PCT, and IL-6/in group D were 5.68 mg/mL, 13.7 pg/mL, and 20.3 ng/, respectively, which were significantly lower than those in groups A, B, and C (*P* < 0.05).

### 3.8. Patient Satisfaction Evaluation

The study investigated the satisfaction of four groups of patients.  Figure 11 shows that the scores of groups A, B, C, and D were 5.28, 7.02, 6.74, and 8.92, respectively. The satisfaction score of group D was significantly higher than that of other groups, and the difference was statistically significant (*P* < 0.05).

## 4. Discussion

Pressure ulcer is a refractory common clinical complication that seriously affects the daily life of patients [21]. Dressing change is a traditional way of treatment, which is unsatisfactory and time-consuming [22]. At present, VSD or PRP treatment is commonly used in clinical practice, in which VSD can provide sufficient nutrition for the wound surface through continuous negative pressure drainage to promote local blood circulation; PRP contains a variety of high concentrations of cytokines and growth factors, and the platelet-rich gel formed by PRP and calcium can effectively stimulate platelets to release a large number of growth factors and then promote the growth and recovery of wound tissue [23, 24]. Kim et al. [25] used a convolutional neural network for low-dose CT image denoising, and the result showed that the convolutional neural network had better high resolution at all dose and contrast levels. Therefore, this study proposes a CT image noise reduction algorithm based on Dr-CNN network model, three algorithms were compared as follows: LDCT, TV, and DNCNN, and were used to evaluate PRP combined with VSD treatment in pressure ulcer. The results revealed that the mean PSNR and SSIM of Dr-CNN network model were 37.21 ± 1.09 dB and 0.925 ± 0.01, respectively, which were higher than those of LDCT, TV, and DNCNN; the mean RMSE and NMAD of Dr-CNN network model were 0.022 ± 0.002 and 0.126 ± 0.012, respectively, which were significantly lower than those of other algorithms, and the differences were statistically significant (*P* < 0.05), indicating that the Dr-CNN network model had better stability and noise reduction effect. In addition, the average running time of the algorithms was compared, and it was found that Dr-CNN network model took longer to process a graph, which may be related to the complexity of the algorithm results and the parameter counts.

A total of 84 subjects were enrolled in the study and randomly divided into groups A, B, C, and D. Each group had different treatment methods. There was no significant difference in the general clinical data among the four groups, indicating the feasibility of the study. In the 84 subjects, 44 cases (52.38%) recovered after treatment, 24 (28.57%) had no change in stage, and pressure ulcer occurred in 16 cases (19.04%). There was no significant difference in the pain scores among the four groups before operation, and the pain scores of groups B, C, and D after operation were significantly lower than those before operation, and the difference had statistical significance. The postoperative pain score of group D was significantly lower than that of other groups, and the differences had statistical significance (*P* < 0.05). It shows that the effect of conventional treatment on relieving the pain of patients is not obvious, although the use of PRP or VSD can relieve the pain, the effect is less than the combination of the two. Liu et al. [26] evaluated the efficacy of PRP gel in the treatment of refractory pressure injury and its effect on wound healing time and patients' quality of life, and the results were similar to this study. The time of complete wound healing in group D was 24.5 ± 2.32 days, which was significantly shorter than that in groups A, B, and C, and the difference had statistical significance (*P* < 0.05). The use of PRP combined with VSD can effectively shorten the wound healing time of patients. On the other hand, the study compared the serum inflammatory factors 20 days after surgery in the four groups. The results showed that there was no great difference in the mean CRP (mg/mL), PCT (pg/mL), and IL-6 (ng/L) values of the four groups of patients before surgery. Postoperative CRP, PCT, and IL-6/in group D were 5.68 mg/mL, 13.7 pg/mL, and 20.3 ng/, respectively, which were significantly lower than those in groups A, B, and C (*P* < 0.05). The results were similar to those of Wang et al. [27]. Finally, the study investigated the satisfaction rate of patients in the four groups. The results suggested that the scores of groups A, B, C, and D were 5.28, 7.02, 6.74, and 8.92, respectively. It could be observed that the satisfaction rate of group D was significantly higher than that of other groups, and the difference had statistical significance (*P* < 0.05).

## 5. Conclusion

In order to explore the clinical efficacy and serum factor level of CT evaluation of PRP combined with VSD based on intelligent algorithm in the treatment of pressure ulcer patients, a CT image denoising algorithm based on Dr-CNN network model was proposed, and the effects of four treatment methods were compared. The results showed that the Dr-CNN network model had the best stability and noise reduction effect, and PRP combined with VSD was effective in the treatment of pressure ulcers. However, this study is a small sample and cannot effectively reflect the overall characteristics. In the later exploration, the number of cases should be increased, the number of samples should be expanded, and the error should be reduced. In general, PRP combined with VSD can effectively relieve the pain of patients and shorten the wound healing time, which is worthy of clinical promotion.

## Figures and Tables

**Figure 1:** Dr-CNN network model.

**Figure 2:** Dr-CNN network structure.

**Figure 3:** Comparison of noise reduction performance of the four algorithms. ((a) PSNR; (b) SSIM; (c) RMSE; (d) NMAD). Note: ^∗^Statistically significant compared with other algorithms (*P* < 0.05).

**Figure 4:** Comparison of average running time of four algorithms.

**Figure 5:** Comparison of noise reduction effect of four algorithms.

**Figure 6:** Comparison of general clinical data of patients.

**Figure 7:** Treatment outcome statistics.

**Figure 8:** Preoperative and postoperative pain scores. (preoperative pain score in (a) and postoperative pain score in (b)). Note: ^∗^The difference had statistical significance relative to other groups (*P* < 0.05).

**Figure 9:** Comparison of postoperative wound healing time. Note: ^∗^Meant a significant difference compared to other groups (*P* < 0.05).

**Figure 10:** Comparison of serum inflammatory factors before and 20 days after operation. ((a) CRP, (b) PCT, and (c) IL-6). Note: ^∗^The difference had statistical significance compared with other groups (*P* < 0.05).

**Figure 11:** Comparison of patient satisfaction.

## Data Availability

The data used to support the findings of this study are available from the corresponding author upon request.
